# Accuracy of Magnetic Resonance Imaging in Diagnosing Placenta Accreta: A Systematic Review and Meta-Analysis

**DOI:** 10.1155/2022/2751559

**Published:** 2022-08-26

**Authors:** Huien Lin, Li Li, Yi Lin, Wenhuan Wang

**Affiliations:** ^1^Department of Medical Imaging, Haikou Maternal and Child Health Hospital, Haikou 570203, China; ^2^Department of Imaging, Hainan Women and Children's Medical Center, Haikou 570216, China

## Abstract

**Background:**

The disease burden and incidence of placenta accreta are increasing worldwide. The morbidity and mortality associated with undiagnosed placenta accreta are both high, highlighting the important of early diagnosis and intervention. In recent years, increasing studies are exploring the diagnostic value of magnetic resonance imaging (MRI) for placenta accreta. Compared with traditional ultrasound, MRI has the advantages of high-resolution, multiangle imaging, and less influence by amniotic fluid and intestinal gas. However, the reported diagnostic accuracy among studies was inconsistent. Therefore, this study is aimed at exploring the diagnostic value of MRI for placenta accreta by systematic review and meta-analysis.

**Methods:**

Relevant literature were systematically searched in PubMed, Ovid, Embase, ScienceDirect database, CNKI, and Wanfang database by using medical subject headings and relevant diagnostic terminologies such as sensitivity, specificity, likelihood ratio, receiver-operating characteristic curve, and area under the curve. The sensitivity, specificity, positive likelihood ratio, negative likelihood ratio, and area under the curve of the included literature were analyzed using stata 17.0 software. Publication bias of the included studies was assessed by Deek's funnel plot. Cochrane *Q* statistics and *I*^2^ statistics were used to test the heterogeneity.

**Results:**

A total of 10 primary publications, comprising 4 retrospective studies and 6 prospective studies, were included in this meta-analysis. The gestational weeks of pregnant women ranged from 32 to 35 weeks, and the sample size ranged from 37 cases to 575 cases. Only 4 studies used the blind method in the process of clinical diagnosis by MRI. The combined sensitivity, specificity, and area of curve under summary receiver-operating characteristic for the diagnosis of placenta accreta by MRI were 0.88 (95% CI, 0.79-0.93), 0.79 (95% CI, 0.68-0.87), and 0.91 (95% CI, 0.88.-0.93), respectively. The combined positive likelihood ratio, negative likelihood ratio, diagnostic odds ratio, and diagnostic score were 4.17 (95% CI, 2.62-6.66), 0.16 (95% CI, 0.09-0.29), 26.61 (95% CI, 10.22-69.28), and 3.28 (95% CI, 2.32-4.24), respectively. No publication bias was noted.

**Conclusion:**

Diagnosis of placenta accreta by MRI has good accuracy and predictive value that warrants clinical promotion.

## 1. Introduction

Placenta accreta spectrum (PAS) refers to the abnormal attachment of placental trophoblasts to the uterine myometrium that can be further divided into placenta accreta, placenta increta, and placenta perforata based on the depth of invasion of the myometrium [1, 2]. Risk factors for PAS mainly include advanced maternal age, cesarean section, scarred uterus, placenta previa diagnosed before delivery, uterine lesions, and assisted reproductive technology. The primary pathophysiological mechanism of placenta accreta may be related to a specific or a combination of factors, such as basal decidua loss, abnormal local oxygen tension, excessive trophoblast invasion, and abnormal vascular remodeling [3, 4]. With the increase in abortion and cesarean section rates, the incidence of placenta accreta has shown an increasing trend worldwide. A recent multicenter Chinese population-based study showed that the incidence of placenta accreta in China had increased from 0.03% in 1980 to 2.2% in 2022, which was higher than in the coastal areas than that in inland areas. Furthermore, the prevalence in developed regions was higher than that in underdeveloped areas in central and western China [5]. Studies have shown that the perinatal mortality of placenta accreta is about 7% [6], while about 50-60% of placenta accreta is not diagnosed before delivery [7, 8]. Due to the increasing disease burden, early diagnosis of placenta accreta is essential for decreasing maternal mortality or morbidity.

Doppler ultrasound is currently the primary imaging technique for diagnosing placenta accreta thanks to its noninvasiveness, economic advantage, and wide availability. However, its diagnostic yield for placenta accreta is adversely influenced by amniotic fluid, intestinal gas, and placental position [8]. In recent years, magnetic resonance imaging (MRI) has been increasingly adopted in the diagnosis of prenatal placental implantation in the realization of its advantages of high-resolution, multiangle imaging, and limited influence by amniotic fluid and intestinal gas [6]. Previous Chinese and English literature have reported the diagnostic accuracy of MRI for placenta accreta with inconsistent sensitivity and specificity. Therefore, a meta-analysis can obtain a more reliable conclusion by systematically combining the indicators of diagnostic accuracy of included studies. Thus, the purpose of this study is to assess the clinical value of MRI for the diagnosis of placenta accreta by systematic review and meta-analysis of published diagnostic studies.

## 2. Methods

### 2.1. Retrieval Strategy

In this study, the following Medical Subject Headings (MeSH) were used in PubMed, Ovid, Embase, ScienceDirect databases, CNKI, and Wanfang databases, respectively, from inception to April 2022: (“placenta accreta” OR “Accreta, placenta” OR “placenta increta” OR “placenta percreta”) AND (“MRI”, “magnetic resonance imaging”) AND (“diagnosis” OR “diagnostic accuracy” OR “sensitivity” OR “specificity”). The database was supplemented and improved by screening other relevant unpublished literature, meeting notes, and contacting experts in relevant clinical fields. The literature screening process is shown in Figure 1 per the PRISMA guideline.

### 2.2. Inclusion and Exclusion Criteria

Retrieved publications were subject to the inclusion and exclusion criteria established below. Inclusion criteria are (1) MRI was used to assist in the diagnosis of placenta accreta in pregnant women with a history of cesarean section or placenta previa; (2) the sample size should be at least 8 cases per group; (3) indicators of true positive (TP), false positive (FP), false negative (FN), and true negative (TN) required for the combined effect value could be calculated directly or indirectly according to the data of the original study; and (4) the diagnosis of placenta accreta was established by histopathological analysis.

Exclusion criteria are (1) academic review, academic conference, review, and case report; (2) the data provided by the article was not enough to calculate the diagnostic accuracy; (3) withdrawn articles; (4) the research content was irrelevant to this study; and (5) publications with study population overlap.

### 2.3. Documentation and Evaluation

The following data were extracted from the included studies two independent researchers: author, publication time, study design (prospective or retrospective), demographic characteristics of the study population (gestational age), sample size, TP, FP, FN, TN, sensitivity, specificity, and the diagnostic gold standard. Discrepancies between the 2 investigators were settled by discussion or consulting with a third investigator. The methodological quality and risk bias of the included studies were assessed by the Quality Assessment of Diagnostic Accuracy Studies (QUADAS), which assessed a total of 14 items phrased as questions that evaluated the disease spectrum, the interpretability of the examination results, whether the blind method was used in the implementation of the trial, the use of the gold standard, the disease progress, the evaluation bias, the combined bias, and the rationality of the included cases.

### 2.4. Statistical Methods

In this study, STATA17.0 (MP) was used for statistical calculation. The relevant diagnostic accuracy indicators, including sensitivity, specificity, diagnostic odds ratio (DOR), negative likelihood ratio, and positive likelihood ratio, were pooled. The summary receiver-operating characteristic (SROC) curves were used to calculate the area under the curve (AUC) of the combined model. The heterogeneity among the included studies was quantified using the Cochrane *Q* statistics and *I*^2^ statistics. When the *I*^2^ statistic exceeded 50%, the random-effect model based on the Dersimonian-Laird method was used to merge the diagnostic accuracy indicators when the *I*^2^ statistic >50%. Otherwise, the Mantel-Haenszel's fixed-effect model was used. Publication bias of the included studies was assessed by Deek's funnel plot. All hypothesis tests were statistically significant with two-sided *P* < 0.05.

## 3. Results

### 3.1. Search Results

A total of 421 relevant literature were generated through the systematic search. After screening according to the inclusion/exclusion criteria, a total of 10 publications [9–18] were included in this meta-analysis, including 4 retrospective studies and 6 prospective studies. The gestational weeks of pregnant women ranged from 32 to 35 weeks, and the sample size ranged from 37 cases to 575 cases. Among the 10 publications, only 4 studies used a blind method in the process of clinical diagnosis with MRI. The characteristics of the included studies are shown in Table 1.

### 3.2. Literature Quality Evaluation

The MIDAS command in STATA 17.0 MP was used to draw a segmented bar chart containing the evaluation criteria of each QUADAS [19]. As shown in Figure 2, the overall quality of the included literature was high. Most of the included literature described the gold standard used, the diagnostic criteria for placenta accreta, and the demographic characteristics and related risk factors for study population. However, most studies included a small sample size, and less than half of the studies used a blind method in diagnosing placenta accreta using MRI.

### 3.3. Meta-Analysis of the Accuracy of MRI in Diagnosing Placenta Accreta

#### 3.3.1. Heterogeneity Analysis

The results indicated high heterogeneity (*Q* = 8.131, *I*^2^ = 75.95%), for which the random-effects model was used to combine the effect sizes. In addition, the sensitivity, specificity, positive likelihood ratio, negative likelihood ratio, and *I*^2^ of the diagnostic odds ratio were all >50%.

#### 3.3.2. Combined Effect Analysis

The pooled sensitivity, specificity, and AUC were 0.88 (95% CI: 0.79-0.93), 0.79 (95% CI: 0.68-0.87), and 0.91 (95% CI, 0.88.-0.93), respectively. The combined diagnostic odds ratio, positive likelihood ratio, negative likelihood ratio, and diagnostic score were 26.61 (95% CI, 10.22-69.28), 4.17 (95% CI, 2.62-6.66), 0.16 (95% CI, 0.09-0.29), and 3.28 (95% CI, 2.32-4.24), respectively (Figures 3–6). The scatter plot of the likelihood ratios showed that the pooled estimates with 95% confidence interval were located in the lower right quadrant, suggesting that the combined accuracy of MRI for diagnosing placenta accreta was poor (Figure 7).

#### 3.3.3. Fagan Nomogram Analysis

A 50% predicted probability was assessed to simulate a clinical situation, resulting in a posttest probability of 81% for a positive test result, while the negative likelihood ratio was 0.16, and the negative posttest probability was 14% (Figure 8).

### 3.4. Publication Bias

The Deek funnel plot (Figure 9) showed a slope coefficient of 0.611, indicating that there was no publication bias in the included studies.

## 4. Discussion

This study showed that MRI has good accuracy in diagnosing placenta accreta. Depending on the degree of myometrial invasion [20], placenta accreta is associated with life-threatening complications that include maternal bleeding, uterine perforation, or even death [21, 22]. Studies have shown that placenta accreta accounted for roughly 1/3 to 1/2 of postpartum emergency hysterectomy [20]. Common risk factors for placenta accreta include advanced maternal age (≥35 years), assisted reproductive technology [6, 23], placenta previa, history of uterine injury, Asherman's syndrome, abnormal uterine anatomy, or uterine pathological status (such as bicornate uterus, adenomyosis, and submucosal myoma) [21]. An apparent dose-response relationship between the frequency of cesarean section and the incidence of placenta accreta has also been noted, as exemplified by the fact that the risk of placenta accreta at the first cesarean section is only 3% [24], which increases to an astonishing 40-67% at 3^rd^ to fifth cesarean section [25]. Epidemiological studies showed accompanying cesarean section rate increase in China [26], and the incidence of placenta accreta had also increased from 0.25/1000 in 1970 [27] to 0.79/1000 in 2003 [28] and 1/533 in 2015 [29]. Although ultrasound [30] is the preferred imaging method for the clinical diagnosis of suspected placental implantation, Aitken et al. have shown that MRI has obvious advantages over ultrasound in predicting the depth of placental implantation and invasion of the surrounding tissue [31]. Furthermore, Bakri et al. [32] and Thorp et al. [33] also suggested that even though ultrasound diagnosis had the advantages of economy and convenience that supports its utility as the mainstream diagnostic technique for placental implantation in the future, MRI has superior diagnostic performance for pathologies of the posterior placenta, thanks to its higher resolution and multiangle imaging of soft tissue that can clearly depict the adjacent anatomical position and vascular distribution during placenta implantation. In addition, MRI can provide more reference information for cesarean section that helps to reduce the risk of intraoperative bleeding. Thus, MRI can still be used as an auxiliary diagnostic method even when ultrasound has clearly diagnosed placenta accreta [34, 35]. However, the imaging signs of placenta accreta by MRI also partially coincide with those of normal pregnant women, such as thinning of the myometrium, uneven signals in the placenta, and blurring of the placenta myometrium junction. The respiratory movement of the fetus and pregnant women may also cause artifact interference to the image quality, which greatly increases the false negative or false positive results of MRI interpretation. Some researchers believe that MRI suffers from several safety and ethical problems, such as long scanning time, annoying scanning noise, and heavy abdominal coil. Therefore, ultrasound is still recommended as the first-line imaging modality for placenta implantation [36].

This study suffers from several limitations. First, most of the included studies did not report the risk factors and baseline characteristics of placenta accreta before the study. Most of the study population was not randomized, which might introduce bias to the present meta-analysis. Second, there was no unified imaging standard for the diagnosis of placenta accreta by MRI. The interpretations of MRI images may be subject to the reader's experience, which may explain the differences in the sensitivity and specificity of placenta accreta diagnosis by MRI reported. Third, this study excluded publications published in languages other than English and Chinese, which may introduce bias on the true diagnostic value of MRI for placenta accreta. However, we believe that this bias should be relatively small since no publication bias was observed in this study. At last, the fact that less than 4 studies were available for each country rendered subgroup analysis at the regional level difficult. Regional differences was considered to be the most likely source of heterogeneity among studies.

## 5. Conclusion

This study showed that MRI had good diagnostic accuracy for diagnosing prenatal placenta accreta. However, due to insufficient evidence for the economic benefit between ultrasound and MRI and considerable differences in imaging diagnostic criteria, it is still recommended to take ultrasound as the first-line imaging modality for placenta accreta. Nonetheless, MRI as an auxiliary imaging modality can still supplement clinical useful information.

## Figures and Tables

**Figure 1:** PRISMA flowchart of literature screening.

**Figure 2:** Sectional bar chart of literature quality evaluation summary by diagnostic experimental research quality evaluation scale tool.

**Figure 3:** Combined sensitivity and specificity forest plot. (a) Combined sensitivity forest map. (b) Combined specificity forest plot.

**Figure 4:** Summary receiver-operating characteristic and the area under the curve after combination.

**Figure 5:** Forest plot for likelihood ratio after combination (LR+, LR-).

**Figure 6:** Forest plot for diagnostic odds ratio and diagnostic score after combination.

**Figure 7:** Distribution scatter diagram of the likelihood ratio (LR+/LR-) of each study and combined estimated value.

**Figure 8:** Fagan nomogram of the accuracy of MRI in the diagnosis of placenta accrete.

**Figure 9:** Deek funnel plot showing publication bias.

**Table 1:** Characteristics of documents included in the analysis.

Included studies	Mean gestational weeks	Sample size	TP	FP	FN	TN	Literature type	Whether the blind method was used
Yan et al. (2022) [18]	33.3 ± 4.6	47	16	3	4	31	Prospective study	No
Riteau et al. (2014) [17]	34 ± 4.7	42	16	25	5	25	Retrospective study	Yes
Maher et al. (2014) [16]	32.4 ± 4.3	575	42	160	7	533	Prospective study	No
Lopes et al. (2019) [15]	35.4 ± 1.1	37	16	28	1	21	Retrospective study	Yes
Elhawary et al. (2013) [11]	33.1 ± 5.1	39	8	5	1	31	Prospective study	No
Ding et al. (2021) [14]	32.92 ± 4.1	89	17	8	2	72	Prospective study	Yes
Einerson et al. (2020) [13]	34.8 ± 4.1	68	44	10	23	24	Prospective study	Yes
Ayati et al. (2017) [12]	32.1 ± 3.98	82	24	12	8	58	Retrospective study	No
Zhang et al. (2021) [10]	34.51 ± 3.19	128	101	3	3	27	Prospective study	Yes
Xiao et al. (2027) [9]	33.29 ± 5.72	150	58	18	2	92	Retrospective study	No

## Data Availability

The data used and analyzed during the current study are available from the corresponding author.

## References

[1] Usta I. M., Hobeika E. M., Abu Musa A. A., Gabriel G. E., Nassar A. H. (2005). Placenta previa-accreta: risk factors and complications. *American Journal of Obstetrics and Gynecology*.

[2] Jauniaux E., Ayres-de-Campos D., Langhoff-Roos J. (2019). FIGO classification for the clinical diagnosis of placenta accreta spectrum disorders,. *International Journal of Gynecology & Obstetrics*.

[3] Silver R. M., Branch D. W. (2018). Placenta accreta spectrum. *New England Journal of Medicine*.

[4] Carusi D. A. (2018). The placenta accreta spectrum: epidemiology and risk factors. *Clinical Obstetrics and Gynecology*.

[5] Mogos M. F., Salemi J. L., Ashley M., Whiteman V. E., Salihu H. M. (2016). Recent trends in placenta accreta in the United States and its impact on maternal–fetal morbidity and healthcare-associated costs, 1998–2011. *The Journal of Maternal-Fetal & Neonatal Medicine*.

[6] Baughman W. C., Corteville J. E., Shah R. R. (2008). Placenta accreta: spectrum of US and MR imaging findings. *Radiographics*.

[7] Mulla B. M., Weatherford R., Redhunt A. M. (2019). Hemorrhagic morbidity in placenta accreta spectrum with and without placenta previa. *Archives of Gynecology and Obstetrics*.

[8] Esakoff T. F., Sparks T. N., Kaimal A. J. (2011). Diagnosis and morbidity of placenta accreta. *Ultrasound in Obstetrics & Gynecology*.

[9] Fang X., Ying X., Aijun T., Haiyan K. (2017). The diagnostic value of ultrasound and MRI in placenta accreta. *China Physician Journal*.

[10] Xiangchen Z., Yingjie H., Jing Y., Zhang Y., He Y. (2021). MRI and ultrasound diagnosis of placenta accreta and their therapeutic evaluation value. *Biomedical Engineering and Clinical*.

[11] Elhawary T. M., Dabees N. L., Youssef M. A. (2013). Diagnostic value of ultrasonography and magnetic resonance imaging in pregnant women at risk for placenta accreta. *The Journal of Maternal-Fetal & Neonatal Medicine*.

[12] Ayati S., Pourali L., Pezeshkirad M. (2017). Accuracy of color Doppler ultrasonography and magnetic resonance imaging in diagnosis of placenta accreta: a survey of 82 cases. *International Journal of Reproductive BioMedicine*.

[13] Einerson B. D., Rodriguez C. E., Silver R. M., Donnelly M. A., Kennedy A. M., Woodward P. J. (2021). Accuracy and interobserver reliability of magnetic resonance imaging for placenta accreta spectrum disorders. *American Journal of Perinatology*.

[14] Ding X., Cao Y., Sun F., Ma A., Zhang F. (2021). Clinical analysis of improved particle swarm algorithm-based magnetic resonance imaging diagnosis of placenta accreta. *Contrast Media & Molecular Imaging*.

[15] Lopes E. S., Feitosa F. E. L., Brazil A. V. (2019). Assessment of sensitivity and specificity of ultrasound and magnetic resonance imaging in the diagnosis of placenta accreta. *Revista Brasileira de Ginecologia e Obstetrícia*.

[16] Maher M. A., Abdelaziz A., Bazeed M. F. (2013). Diagnostic accuracy of ultrasound and MRI in the prenatal diagnosis of placenta accreta. *Acta Obstetricia et Gynecologica Scandinavica*.

[17] Riteau A.-S., Tassin M., Chambon G. (2014). Accuracy of ultrasonography and magnetic resonance imaging in the diagnosis of placenta accreta. *PLoS One*.

[18] Yan G., Liao Y., Li K. (2022). Diffusion MRI based myometrium tractography for detection of placenta accreta spectrum disorder. *Journal of Magnetic Resonance Imaging*.

[19] Whiting P. F., Weswood M. E., Rutjes A. W. S., Reitsma J. B., Bossuyt P. N. M., Kleijnen J. (2006). Evaluation of QUADAS, a tool for the quality assessment of diagnostic accuracy studies. *BMC Medical Research Methodology*.

[20] Leyendecker J. R., DuBose M., Hosseinzadeh K. (2012). MRI of pregnancy-related issues: abnormal placentation. *American Journal of Roentgenology*.

[21] Fadl S., Moshiri M., Fligner C. L., Katz D. S., Dighe M. (2017). Placental imaging: normal appearance with review of pathologic findings. *Radiographics*.

[22] Parra-Herran C., Djordjevic B. (2016). Histopathology of placenta creta: chorionic villi intrusion into myometrial vascular spaces and extravillous trophoblast proliferation are frequent and specific findings with implications for diagnosis and pathogenesis. *International Journal of Gynecological Pathology*.

[23] Qiong Z., Shengli L. (2013). New progress in prenatal diagnosis of placenta accreta. *Chinese Journal of Medical Ultrasound: Electronic Edition*.

[24] Getahun D., Oyelese Y., Salihu H. M., Ananth C. V. (2006). Previous cesarean delivery and risks of placenta previa and placental abruption. *Obstetrics & Gynecology*.

[25] Clark S. L., Koonings P. P., Phelan J. P. (1985). Placenta previa/accreta and prior cesarean section. *Obstetrics and Gynecology*.

[26] Li H.-T., Luo S., Trasande L. (2017). Geographic variations and temporal trends in cesarean delivery rates in China, 2008-2014. *JAMA*.

[27] Miller D. A., Chollet J. A., Goodwin T. M. (1997). Clinical risk factors for placenta previa-placenta accreta. *American Journal of Obstetrics and Gynecology*.

[28] Cheng K. K., Lee M. M. (2015). Rising incidence of morbidly adherent placenta and its association with previous caesarean section: a 15-year analysis in a tertiary hospital in Hong Kong. *Hong Kong Medical Journal*.

[29] Wu S., Pickett K., Hibbard J. (2003). Abnormal placentation: where are we now? Analysis of the last twenty years. *American Journal of Obstetrics & Gynecology*.

[30] Jauniaux E. R. M., Alfirevic Z., Bhide A. G. (2019). Placenta praevia and placenta accreta: diagnosis and management: green-top guideline no. 27a. *BJOG*.

[31] Aitken K., Allen L., Pantazi S. (2016). MRI significantly improves disease staging to direct surgical planning for abnormal invasive placentation: a single centre experience. *Journal of Obstetrics and Gynaecology Canada*.

[32] Bakri Y. N., Rifai A., Legarth J. (1993). Placenta previa-percreta: magnetic resonance imaging findings and methotrexate therapy after hysterectomy. *American Journal of Obstetrics & Gynecology*.

[33] Thorp J. M., Councell R. B., Sandridge D. A., Wiest H. H. (1992). Antepartum diagnosis of placenta previa percreta by magnetic resonance imaging. *Obstetrics and Gynecology*.

[34] Committee on Obstetric Practice (2012). Committee opinion no. 529: placenta accreta. *Obstetrics and Gynecology*.

[35] Kilcoyne A., Shenoy-Bhangle A. S., Roberts D. J., Sisodia R. C., Gervais D. A., Lee S. I. (2017). MRI of placenta accreta, placenta increta, and placenta percreta: pearls and pitfalls. *American Journal of Roentgenology*.

[36] Jauniaux E., Bhide A. (2017). Prenatal ultrasound diagnosis and outcome of placenta previa accreta after cesarean delivery: a systematic review and meta-analysis. *American Journal of Obstetrics and Gynecology*.

